# An ileal gastrointestinal stromal tumor misdiagnosed as pelvic metastases from rectal cancer: a case report

**DOI:** 10.3389/fonc.2023.1164391

**Published:** 2023-04-25

**Authors:** Jun Ma, Juan Zhu, Shuihong Yu, Chaoping Zhou, Shuqiang Duan, Yaming Zhang

**Affiliations:** ^1^ Department of General Surgery, Anqing Municipal Hospital, Anqing, China; ^2^ Department of Imaging, Anqing Municipal Hospital, Anqing, China; ^3^ Research and Experimental Center, Anqing Medical and Pharmaceutical College, Anqing, China; ^4^ Department of Pathology, Anqing Municipal Hospital, Anqing, China

**Keywords:** rectal cancer, GIST, synchronous tumors, surgery, metastases

## Abstract

With the advancement of imaging and pathological diagnostic methods, it is not uncommon to see synchronous gastrointestinal stromal tumors (GIST) and other primary cancers, the most common of which are synchronous gastric cancer and gastric GIST. However, synchronous advanced rectal cancer and high-risk GIST in the terminal ileum are extremely rare, and they are easily misdiagnosed as rectal cancer with pelvic metastases due to their special location near iliac vessels. Herein, we report a 55-year-old Chinese woman with rectal cancer. Preoperative imaging revealed a middle and lower rectal lesion with a right pelvic mass (considered possible metastasis from rectal cancer). Through multidisciplinary discussions, we suspected the possibility of rectal cancer synchronous with a GIST in the terminal ileum. Intraoperative exploration by laparoscopy revealed a terminal ileal mass with pelvic adhesion, a rectal mass with plasma membrane depression, and no abdominal or liver metastases. Laparoscopic radical proctectomy (DIXON) plus partial small bowel resection plus prophylactic loop ileostomy was performed, and the pathological report confirmed the coexistence of advanced rectal cancer and a high-risk ileal GIST. The patient was treated with the chemotherapy (CAPEOX regimen) plus targeted therapy(imatinib) after surgery, and no abnormalities were observed on the follow-up examination. Synchronous rectal cancer and ileal GIST are rare and easily misdiagnosed as a rectal cancer with pelvic metastases, and careful preoperative imaging analysis and prompt laparoscopic exploration are required to determine the diagnosis and prolong patient survival.

## Background

Multiple synchronous primary malignancies are defined as two or more primary tumors that are each diagnosed at an interval of less than 6 months apart (1). Among patients with synchronous gastrointestinal stromal tumors (GIST) and malignant epithelial tumors, synchronous gastric or esophageal cancer and gastric GIST are the most common (2–4); however, there have also been scattered reports of synchronous rectal cancer and rectal GIST (5, 6), synchronous colon cancer and intestinal GIST (7, 8), or synchronous breast cancer and GIST (9). However, synchronous rectal cancer and ileal GIST are extremely rare, ileal GIST located in the pelvic easily misdiagnosed as metastatic lesions from rectal cancer.

Herein, we report an extremely rare case of advanced rectal cancer synchronous with a high-risk GIST of the terminal ileum that was diagnosed and treated by preoperative and intraoperative assessments.

## Case presentation

A 55-year-old Chinese woman had blood in her stool without any obvious cause since 1 month prior. The patient had no abdominal pain or distension, no chills or fever, no anal pain, a normal diet and sleep, normal urine, and no significant weight loss during the course of the disease. The patient was diagnosed with rectal cancer by colonoscopy, and the pathology results suggested adenocarcinoma. The patient had a history of hysterectomy for uterine fibroids and decompression for traumatic brain injury. The patient had no history of familial cancer.

No enlarged lymph nodes were found on palpation of the clavicle and groin, the abdomen was flat and soft, and no abnormal masses were palpable. A cauliflower-like hard mass was palpable on the anterior wall of the rectum approximately 4 cm from the anus, in a 1/2 circle around the rectal cavity; the finger could pass but did not touch the upper edge of the mass, and the finger sleeve was blood-stained. The patient’s preoperative hemoglobin level was 100 g/l, her platelet level was 80 × 10^9^/l, and the stool was positive for occult blood. Other parameters were normal.

On March 23, 2022, computed tomography (CT) showed a soft tissue mass on the right side of the pelvis with poorly defined borders and uneven enhancement, and no obvious enlarged lymph nodes were found in the pelvis. The wall of the middle and lower rectum was thickened, and the lumen of the lesion was narrowed, with mild enhancement (**Figures 1A, B**).

**Figure 1:** Preoperative imaging data. **(A)** CT showed the blood supply of the tumor originating from the branches of the SMA (red arrow). **(B)** CT showed a soft tissue mass on the right side of the pelvis (red arrow); the wall of the middle and lower rectum was thickened, with mild enhancement (white arrow). **(C, D)** MRI showed a mass in the pelvis (red arrow); the rectal lesion appeared hyperintense on DWI (white arrow).

On March 25, 2022, magnetic resonance imaging (MRI) showed a mass next to the right iliac vessels, which appeared with isointensity on T1-weighted imaging, slight hyperintensity on T2-weighted imaging, and hyperintensity on T2-weighted fat-suppressed imaging and diffusion-weighted imaging (DWI, b800). Apparent diffusion coefficient (ADC) imaging showed a low signal, and the size of the lesion was determined to be approximately 5.4 cm × 4.9 cm; the boundary was still clear (considering the possibility of metastasis) (**Figure 1C**).

MRI also showed irregular thickening of the rectal bowel wall, which appeared with isointensity on T1-weighted and T2-weighted imaging. DWI (b800) showed a significantly hyperintense signal, with predominantly intraluminal growth of the lesion (**Figures 1C, D**). The tumor was considered as rectal cancer, mesorectal fascia (MRF) showed a negative result, extramural vascular invasion (EMIV) showed a negative result, and the preoperative clinical stage was cT3N0Mx (considering the possibility of ovarian or lateral lymph node metastases).

We suggested positron emission tomography-computed tomography (PET-CT) to help improve the accuracy of diagnosis for adequate preoperative evaluation, but the patient refused PET-CT due to financial reasons. Through multidisciplinary discussions, we suspected the possibility of rectal cancer synchronous with a GIST in the terminal ileum, and the final preoperative clinical stage was cT3N0M0.

On March 28, 2022, the patient underwent laparoscopic exploration under general anesthesia. The patient was placed in lithotomy position, and traditional five-port access of laparoscopic radical proctectomy with CO_2_ insufflation of abdominal space (pressures of 12 mmHg) was performed. We found no ascites in the abdominal cavity and no metastatic nodules in the peritoneum, greater omentum, or liver. At a distance of 80 cm from the ileocecal valve, a small intestinal mass of approximately 6 cm in size was observed with an uneven epidermis and a rich blood supply, which was adherent to the pelvic cavity (**Figure 2A**). We loosened the adhesion between the small bowel tumor and the pelvic cavity (**Figures 2B, C**) and placed the tumor in the right paracolic sulcus. A distinct depression was visible in the anterior wall of the rectum, which was the location of the rectal lesion (**Figure 2D**). We considered the possibility of rectal cancer synchronous with a GIST in the terminal ileum, and laparoscopic radical proctectomy (DIXON) plus partial small bowel resection was performed.

**Figure 2:** Surgical procedure. **(A)** A small intestinal mass with a rich blood supply was adherent to the pelvic cavity(white arrow). **(B, C)** The adhesion between the small bowel tumor(white arrow) and the pelvic cavity was loosened. **(D)** A distinct depression was visible in the anterior wall of the rectum, which was the location of the rectal lesion (white arrow). **(E, F)** The roots of the interior mesenteric artery (IMA) were dissected under laparoscopy, and the central lymph nodes were cleared. **(G)** The rectum was excised with a 60-mm linear-stapler (one firing) 2 cm below the tumor. **(H)** End-to-end anastomosis of the rectal stump and sigmoid colon was performed.

The roots of the interior mesenteric artery (IMA) were dissected under laparoscopy, and the central lymph nodes were cleared (**Figure 2E, F**). After freeing the rectum from the surrounding space and coping with the rectal mesentery, the rectum was excised with a 60-mm linear stapler (one firing) 2 cm below the tumor (**Figure 2G**) .

A 5-cm median incision was made below the umbilicus, and the specimen was removed. The staple holder was placed into the sigmoid colon and repositioned into the abdominal cavity. The ileal tumor was lifted using a subumbilical incision, and after partial resection of the small bowel, lateral anastomosis was performed.

Subsequently, the small bowel was placed into the abdominal cavity, the pneumoperitoneum was reestablished, and end-to-end anastomosis of the rectal stump and sigmoid colon was performed with a 29-mm circular stapler (**Figure 2H**). A prophylactic loop ileostomy was created to reduce the possibility of postoperative anastomotic leakage.

The patient recovered well and was discharged 10 days after the operation.

Postoperative pathological examination of the rectum showed stage IIB (pT4aN0M0), moderately differentiated adenocarcinoma with no lymph node involvement (0/28) (**Figure 3A**). The resection margin and circumferential margin (CRM) showed a negative result. Immunohistochemical marker results were as follows: CK7(-), CK20(+), CDX-2(+), HER-2 (−), p53 (+), Ki-67 (approximately 90%), MSH2 (+), MSH6 (+), MLH1 (+), and PMS2 (+).

**Figure 3:** Photomicrographs. **(A)** Moderately differentiated invasive adenocarcinoma (hematoxylin and eosin, ×20 magnification). **(B)** Small intestinal tumor consisting of fasciculate spindle cells (hematoxylin and eosin, ×40 magnification).

Postoperative pathological examination of the small bowel showed a spindle cell-type stromal tumor 6 cm × 5 cm × 3.5 cm in size (**Figure 3B**), with a mitotic count less than 5/5 mm^2^ and no tumor necrosis; the tumor was high risk, with a WHO prognostic grouping of 3a. The resection margin was negative. Immunohistochemical marker results were as follows: CD117 (+), CD34 (+), Des (-), DOG-1 (+), Ki-67 (1%+), S-100 (-), ALK (-), SMA (-). Genetic testing showed a c-KIT (exon 9) mutation.

Between April 2022 and October 2022, the patient continued adjuvant therapy after surgery, completing eight cycles of CAPEOX regimen (capecitabine plus oxaliplatin) and a half year of targeted therapy (imatinib 400 mg/day), and was suggested to continue targeted therapy for 2.5 years. The patient refused postoperative radiotherapy due to a fear of radiation-related complications. No widespread metastasis or local progression was found in the latest follow-up (**Figure 4**). The timeline is shown in **Table 1**.

**Figure 4:** The latest imaging data. **(A, B)** CT showed no metastatic disease or local progression, and the anastomosis healed well (white arrow).

**Table 1:** The medical history of the patient.

Time series	Diagnosis and treatment details
March 2022	The patient was diagnosed with rectal cancer.
March 23, 2022	The imaging considered rectal cancer with pelvic metastases.
March 26, 2022	Through multidisciplinary discussions, we suspected the possibility of rectal cancer synchronous with a GIST in the terminal ileum.
March 28, 2022	Intraoperative exploration revealed rectal cancer synchronous with a GIST in the terminal ileum, and DIXON plus partial small bowel resection was performed.
April 4, 2022	The patient was discharged, and the pathological report confirmed the coexistence of advanced rectal cancer and a high-risk ileal GIST.
Between April 2022 and October 2022	The patient was treated with the adjuvant chemotherapy plus targeted therapy.
From October 2022 to present	Targeted therapy was continued, and no metastasis or progression was found.

## Discussion

Synchronous advanced rectal cancer and high-risk ileal GIST have not been reported in detail before. Yan-Jun Liu et al. reported only one case of synchronous colorectal cancer and an intestinal GIST among 6,530 cases of colorectal cancer; however, the study did not specify whether it was rectal cancer (1).

In this case, the patient received a clear diagnosis, and treatment was successful. If the patient had been misdiagnosed with rectal cancer and pelvic metastasis and did not promptly undergo laparoscopic exploration and resection, and preoperative neoadjuvant therapy had been performed with a disastrous effect, then the small intestinal GIST would have inevitably progressed. Patients may experience obstruction, bleeding, or even tumor rupture and extensive abdominal metastasis, which significantly reduces patient survival (10–13).

Analyzing the case, possible reasons for the misdiagnosis of this patient are as follows: (1) while the coexistence of rectal cancer and terminal ileal GIST is rare, the diagnosis of advanced rectal cancer in this case was clear, so we might easily suspect that the malignant abdominal lesion may be an metastasis from the rectum; (2) the lesion was located next to the right iliac vessels and had a rich blood supply, so it was not difficult to suppose the possibility of rectal cancer with pelvic metastasis (14).

The key point in the diagnosis of this case was the differentiation between GIST and pelvic metastases from rectal cancer, and imaging examinations including CT or MRI were often performed. First of all, GIST had a round shape, rich blood supply, and clear boundary. Because GIST were often accompanied by intratumor bleeding and central necrosis, they were revealed uneven enhancement (15). Secondly, most pelvic metastases were mainly multiple and their boundaries were unclear and tended to infiltrate the adjacent tissue. MRI with DWI had potential in diagnosing pelvic metastases in patients with rectal cancer (16). Thirdly, on the arterial-phase imaging, several nourishing blood vessels were found in GIST, whereas they were almost undetected in pelvic metastases. Finally, the patient refused PET-CT due to financial reasons that would have been important to help improve the accuracy of diagnosis for adequate preoperative (17).

In this successful case, laparoscopic exploration was promptly performed to determine the diagnosis. This case is enlightening due to the following: (1) When the patients were in normal physical condition, laparoscopic exploration could be used to determine the diagnosis in controversial cases. (2) Through careful review of the imaging findings, we found that the blood supply of the tumor originated from the branches of the superior mesenteric artery (SMA), so the tumor was considered to originate from the small bowel (**Figure 1A**). (3) The incidence of small bowel tumors is low; however, among them, the incidence of stromal tumors is high. The tumor in this case was rounded, with a rich blood supply, and the lesion showed obvious enhancement, which is consistent with the imaging manifestations of gastrointestinal tumors (18, 19).

## Conclusion

In conclusion, the coexistence of advanced rectal cancer and a high-risk ileal GIST is extremely rare and easily misdiagnosed as a rectal cancer with pelvic metastases. Careful preoperative imaging analysis and prompt surgery can prolong the survival of patients.

## Data availability statement

The original contributions presented in the study are included in the article/supplementary material. Further inquiries can be directed to the corresponding author.

## Ethics statement

Written informed consent was obtained from the participant/patient for the publication of this case report.

## Author contributions

All authors read and approved the final manuscript. JM wrote and edited the original draft. JZ and SY contributed to data collection and analysis. SD and CZ reviewed the literature. Y-MZ reviewed the final manuscript. All authors contributed to the article and approved the submitted version.
